# Personalized Intelligent Syndrome Differentiation Guided By TCM Consultation Philosophy

**DOI:** 10.1155/2022/6553017

**Published:** 2022-11-07

**Authors:** Minghuan Li, Guihua Wen, Jiahui Zhong, Pei Yang

**Affiliations:** ^1^South China University of Technology, School of Computer Science and Engineering, Guangzhou 510000, China; ^2^Guangzhou University of Chinese Medicine, Guangzhou 510000, China; ^3^Guangdong Provincial People's Hospital, Guangdong Academy of Medical Sciences, Guangdong Geriatric Institute, Guangzhou 510000, China

## Abstract

Traditional Chinese Medicine (TCM) is one of the oldest medical systems in the world, and inquiry is an essential part of TCM diagnosis. The development of artificial intelligence has led to the proposal of several computational TCM diagnostic methods. However, there are few research studies among them, and they have the following flaws: (1) insufficient engagement with the patient, (2) barren TCM consultation philosophy, and (3) inadequate validation of the method. As TCM inquiry knowledge is abstract and there are few relevant datasets, we devise a novel knowledge representation technique. The mapping of symptoms and syndromes is constructed based on the diagnostics of traditional Chinese medicine. As a guide, the inquiry knowledge base is constructed utilizing the “Ten Brief Inquiries,” TCM's domain knowledge. Subsequently, a corresponding assessment approach is proposed for an intelligent consultation model for syndrome differentiation. We establish three criteria: the quality of the generated question-answer pairs, the accuracy of model identification, and the average number of questions. Three TCM specialists are asked to undertake a manual evaluation of the model separately. The results reveal that our approach is capable of pretty accurate syndrome differentiation. Furthermore, the model's question and answer pairs for simulated consultations are relevant, accurate, and efficient.

## 1. Introduction

Hospitals in China offer plenty of consultations daily and have an imbalanced doctor-patient ratio. With so many patients, doctors work long and exhausting hours, necessitating the development of a quick and effective automated aided consultation mechanism to satisfy patients' immediate requirements while relieving doctor strain. Thousands of years of clinical experience and a solid theoretical framework support traditional Chinese medicine's efficacy [1–6]. Inspection, Auscultation, Inquiry, and Palpation, which are extensively utilized in TCM hospitals in China and worldwide, are the four primary diagnostic techniques employed in TCM hospitals. Of the more than 600 prevalent diseases, more than 75% are acquired through the inquiry since it is a critical way for doctors to comprehend the etiology, course of therapy, and subsequent development of a patient's ailment [7]. Furthermore, TCM has certain norms and guidelines for the content and chronology of the inquiry, and the “Ten Brief Inquiries” is a generalization of it [8]. As a result, TCM consultation is ideal for developing a quick and effective automated auxiliary consultation mechanism.

The term “syndrome” is used in TCM to describe a group of related symptoms that characterize the body's reaction to a disease process and its motions and changes. Four diagnostic techniques are employed to determine the patient's syndromes for follow-up therapy.

As artificial intelligence advances, more research is merging artificial intelligence with medicine. Intelligent diagnosis, based on medical expertise and coupled with artificial intelligence to accomplish autonomous diagnosis, is one of the current hot topics for interdisciplinary study. In the context of intelligent diagnosis in TCM, researchers have completed prescription recommendations and physique identification based on the tongue or facial images (Hu et al. [9], Li et al. [10], Wen et al. [11], Li et al. [12], Liao et al. [13], Hu et al. [14]), feature extraction after sound acquisition (Jiang et al. [15]), and designed pulse feature extraction methods for wrist pulse analysis (Lisheng et al. [16], Zhang et al. [17], Zhang et al. [18]). Inspection, auscultation, olfaction, and palpation can be done with cameras or sensors to collect the necessary signal data, which is analyzed using artificial intelligence algorithms to achieve an intelligent diagnosis. In contrast, inquiry necessitates the doctor to ask questions customized to the patient's circumstances and obtain the essential diagnostic information through several interactions with the patient. Doctors accumulate empirical knowledge from years of clinical practice and establish a diagnosis by intuitively comparing it to comparable instances in the past. This TCM inquiry knowledge is empirical and hazy, making it difficult to extract and communicate. On the other hand, the absence of TCM consultation data precludes the application of deep learning algorithms.

There is limited TCM inquiry research on intelligent diagnosis compared to examination, auscultation, olfaction, and palpation. Furthermore, present intelligent inquiry research lacks patient engagement, does not include TCM consultation philosophy, and has not thoroughly confirmed the efficacy of the proposed methodology. An intelligent diagnosis can acquire various possible syndromes using examination, auscultation, and palpation. However, since more than 75% of symptoms are inferred through inquiry, the candidate syndromes derived from the three diagnoses above must be further identified and verified by inquiring.

In this paper, we use the TCM consultation philosophy to build an intelligent inquiry model that can engage with patients to identify candidate syndromes. There are two current challenges.

(1) The abstract nature of TCM knowledge, which makes it difficult to convert TCM knowledge into a computer-friendly format; (2) the scarcity of TCM consultation data, as no TCM consultation dataset that meets the requirements of deep learning has yet emerged, making it impossible to learn features using deep learning methods. As a result, rather than employ current popular deep learning approaches, we create a novel means of expressing TCM knowledge and present a model of syndrome differentiation (Syndrome Differentiation Model, SDM) to aid doctors in clinical diagnosis. Firstly, the syndromes and symptoms from TCM diagnostic theory and clinical practice are mapped, and question-answer pairs represent symptoms. The inquiry syndrome base and the question base are constructed on this foundation. Secondly, using the Ten Brief Inquiries guide, the question and answer mapping is sorted and ordered to build the inquiry knowledge base. Finally, the SDM is implemented in a client-server architecture. The contributions of this paper are summarized in the following points:

- We innovatively propose a TCM domain knowledge-driven intelligent consultation approach based on ‘Ten Brief Inquiries,' which improves the efficiency of automated consultations while reducing the strain on clinicians.
- In line with the proposed intelligent consultation method, we develop the Syndrome Differentiation Model (SDM), which generates targeted question-answer pairs based on candidate syndromes and interacts with the patient several times to identify the patient's syndromes.
- Using Diagnostic Chinese Medicine and clinical practice, we build the inquiry syndrome base and the question base to skillfully illustrate the relationship between the symptoms, syndromes, and question-answer pairs.

## 2. Related Works

In various medical systems, consultation is frequently utilized as a valuable technique for clinicians to better understand their patients' problems. Because various medical systems have distinct guiding ideas and treatment procedures, the research on intelligent consultation should be conducted individually for each medical system.

Several intelligent consultation studies in Western medicine may generate illness information based on the user's symptoms in a restricted domain. Many online medical consultation records belonging to Western medicine practitioners have appeared on the Web as a result of the development and popularity of the Internet, and some researchers have used these records as a corpus to build a dialogue system that automatically responds to users' medical questions. Shi et al. [19] adopted a label-embedded attention model to apply poorly supervised learning to focus on dispersed medical keywords and perform slot filling on medical conversations. Wei et al. [20] created a dataset based on patient self-reports and doctor-patient interactions on an online medical forum. They suggested a task-oriented dialogue system to capture symptoms other than those reported by the patients. GAMP, a system for automated diagnosis developed by Xia et al. [21], uses the GAN generator as a policy network that motivates the model to choose the most discriminative symptoms for diagnosis. To incorporate domain knowledge into response creation, Li et al. [22] developed a knowledge-oriented multitask Multisource Seq2seq architecture (MSSGK) and three attention methods to offer more suitable response generation guidance. As a result of differences in diagnostic thinking and a lack of data, these methods cannot be directly transferred to TCM.

Inquiry is considered “the key to identifying the condition and the primary job in treating it” in TCM. Due to the absence of inquiry data sets in TCM, there is little research on intelligent consultation compared to Western medicine. Based on their approaches and aims, existing research can be classified into the following categories.

### 2.1. Reasoning-Based Approaches

By creating appropriate reasoning methods, such as case-based reasoning, fuzzy reasoning, a mix of case-based and fuzzy reasoning, and uncertain reasoning about plausibility, reasoning-based approaches simulate the process of syndrome identification. Yang et al. [23] created a case library based on prominent TCM practitioners' treatment experiences and then used case reasoning to replicate the TCM diagnosis process, inferring the likelihood of the patient's syndrome based on symptom information and proposing prescriptions. Zhang et al. [24] categorized symptoms into necessary, necessary and sufficient, probable, and negative symptoms and used fuzzy reasoning and validation mechanisms to get diagnostic judgments. Case inference and fuzzy inference were coupled by Li et al. [25]. For a TCM case, the system conducts case inference first, then moves to the fuzzy mechanism for fuzzy inference if no similar instance is found in the case base. Li and Zong [26] developed an expert system for assisting diagnosis in TCM based on an uncertainty inference model. To create an expert system for TCM software, Zhang [27] wrote inference rules in DRL language based on “ Treatise on Febrile Diseases.”

### 2.2. Deep Learning-Based Approaches

Deep learning in combination with TCM advice is still a relatively new field of study because deep learning is built on data, with a focus on learning from large volumes of data, while data from TCM inquiry is in little supply. The application of artificial neural networks in TCM diagnosis was summarized by Shi and Zhou [28]. TCM diagnosis is considered a mapping process from symptoms to diagnostic outcomes, with quantified instances acting as RNN training samples. The quantified values of symptoms are input to the RNN during diagnosis, and the output is used to calculate the diagnosis result. Ren and Guo [29] gathered TCM cases to construct a structured TCM database, created a multi-label active learning diagnostic classifier, and integrated training using various models, including convolutional neural networks, decision trees, and random forests. There are still issues with these approaches: they are mainly at the experimental stage, the sample sizes utilized are tiny, the methods used to quantify the samples are too simplistic, and they are challenging to interpret.

### 2.3. Template-Based Approach

A template or scale is created in advance for the patient to fill out, and a diagnosis is reached using procedural judgment. Luo and He [7] designed an inquiry software that collects data from a front-end template, makes decisions based on diagnostic criteria from a database management template and then outputs the results. Some research has created TCM syndrome questionnaires and employed questionnaires to collect data on the four diagnoses, which were then classified using clustering and hidden structure model analysis [30].

For the time being, most existing methods are based on disease cases or scales, and no studies have applied the TCM consultation philosophy. In these studies, only one data entry is required and lacks interactivity, meaning patients must describe all their symptoms to get a more accurate diagnosis. However, during the actual diagnostic process, the patient first conveys specific, apparent subjective symptoms to the doctor. Some crucial symptoms are still missed due to inconspicuous subjective feelings, tension, physical discomfort, and other reasons. At this point, the doctor will ask the patient questions for the patient to offer the missing symptoms in time, which provides a reasonable basis for the diagnosis and therapy. Furthermore, the majority of the studies did not evaluate the efficacy of the proposed approaches, and some confirmed the methods' accuracy without manual review.

## 3. Materials and Methods

### 3.1. Diagnosis Framework of TCM

Current TCM diagnosis is somewhat poor in diagnostic localization and quantification due to historical circumstances. Existing Western diagnostic equipment, on the other side, is incompatible with TCM diagnostic therapy and cannot be employed in the area of TCM. TCM diagnostic equipment must be developed using TCM discriminating thinking and the most sophisticated science and technology.

Like other medical disciplines, TCM has a comprehensive theoretical framework, from diagnosis to treatment to therapeutic assessment, all based on its theoretical features, each with its diagnostic form and content, and all consistent with backward and forward treatment theory derivation. TCM takes a holistic approach to understand the human body and illness. Inspection, auscultation, inquiry, and palpation are used to analyze the patient's holistic symptoms before establishing the etiology of the patient's sickness and the kind of syndrome.  Figure 1 depicts the diagnosis framework of TCM.

Internal bodily diseases can be mirrored on the body's surface, according to TCM theory. The patient's self-perception and the doctor's observation of the patient's body surface features are frequently utilized to infer the patient's interior illness in TCM diagnosis and therapy. The aberrant characteristics on the body's surface are observable symptoms, and this approach to diagnosis,“knowing the inside by the surface,” continues to play a significant role in clinical diagnosis in different fields of medicine.

The syndrome, which defines the features of the various stages of the disease, is the diagnostic conclusion in TCM. Because multiple intrinsic lesions may cause the same symptoms to appear and one lesion may cause multiple symptoms to appear, there is a causal relationship between an intrinsic lesion in the body causing observable symptoms, and the opposite is not valid. Every medical science uses symptoms to reason about the probability of disease. Assuming the syndrome or disease is *y*, and the symptom is *x*, Bayes' theorem states that:

(1) $$\begin{array}{c} P\left(y|x\right)=\frac{P\left(x|y\right)P\left(y\right)}{P\left(x\right)}\text{.} \end{array}$$

Knowing the probability *P*(*y*) that patient *p* has illness *y*, the probability *P*(*x*) that patient *p* has symptom *x*, and the probability *P*(*x|y*) that patient *p* has symptom *x* because of disease *y*, the (1) can be used to calculate the probability *P*(*y|x*) that patient *p* has symptom *x* and disease *y*.

TCM diagnosis is based on four diagnostic methods that are used to obtain distinct symptoms from the patient, which are different reflections of the intrinsic lesions of the patient's body, and then reach diagnostic conclusions. Because the same lesion can affect several organs and the symptoms of each organ are complimentary, it is reasonable to combine all four diagnoses. The patient's lesion triggers a variety of symptoms. In view of the fact that the patient's lesion has been determined and the symptoms are exclusively associated with the lesion, we may assume that these symptoms are independent of one another and yield:

(2) $$\begin{array}{c} P\left(y|x_{i}\right)=\frac{P\left(x_{i}|y\right)P\left(y\right)}{P\left(x_{i}\right)}\text{,} \end{array}$$

where *y* is a certain lesion, symptom *x*_*i*_ ∈ *X*, and *X* = {*x*_1_, *x*_2_, ..., *x*_*n*_} represents the set of symptoms of length *n* caused by lesion *y*.

The four diagnostic approaches collect the patient's various symptoms from multiple viewpoints before determining the patient's syndromes utilizing the correlation of all four examinations:

(3) $$\begin{array}{c} P\left(y|s_{1}\cup s_{2}\cup s_{3}\cup s_{4}\right)=\overset{4}{\underset{i=1}{\sum }}P\left(y|s_{i}\right)\text{,} \end{array}$$

where *y* denotes the patient's syndrome and *s*_*i*_(*i* ∈ {1,2,3,4}) denotes the patient's symptoms set as determined by each of the four diagnostic procedures. Each diagnostic approach is independent, and combining the four diagnostic methods is appropriate. The more accurate each diagnostic approach is, the more accurate the probability it calculates and the likelihood of the final combined reference. Consequently, it is prudent to continue enhancing the accuracy of each diagnostic method. In scientific research, we can concentrate on one diagnostic approach, and as long as we enhance its accuracy, the whole diagnostic accuracy will improve when combined.

### 3.2. Proposed Method

#### 3.2.1. Task Description

This paper focuses on the method of inquiry in the diagnostic framework of TCM. Doctors generally first obtain candidate syndromes through inspection, auscultation, and palpation, then determine the content of the consultation based on the candidate syndromes to achieve targeted questions for different patients. TCM has its own set of norms and principles for inquiring, which are part of the body of knowledge in the field of TCM consulting, the most classic being the Ten Brief Inquiries [8]. We aim to develop a model based on the Ten Brief Inquiries to imitate a doctor's consultation. The proposed Syndrome Differentiation Model (SDM) generates targeted questions and answers based on the candidate syndromes to further interact with the patient and ultimately ascertain the patient's actual syndromes. To determine the patient's final syndrome, the model first generates targeted questions and candidate answers based on the candidate syndromes. Then the model interacts with the patient numerous times to learn about their symptoms and compares them with the candidate syndromes, with the most excellent match serving as the patient's final syndrome. The SDM comprises three major parts: an inquiry knowledge base, an inquiry syndrome base, and an inquiry reasoning model.

#### 3.2.2. Knowledge Representation of Inquiry

Questions and candidate answers produced from TCM diagnostic theory and clinical practice are used in the representation, and structuring of TCM inquiry knowledge [31–33]. The mapping of symptoms to syndromes is produced by sorting through the 225 prevalent syndromes according to Chinese medicine's diagnostic science, which is a priori knowledge. It should be noted that the syndrome correlates with symptoms received from the remaining three diagnostic modalities: such symptoms were examined prior to the inquiry. Thus only those gained during the consultation were included in the mapping. We can attain all of the symptoms of a syndrome and vice versa.

During the actual diagnosis procedure, the doctor receives diagnostic information from the patient through a conversation. As a result, a mapping between symptoms and syndromes is established. Symptoms are expressed as question-answer pairs: *z* = (*q, a*), where *z* is the symptom, *q* is the question, and *a* is the answer. The symptoms [fear of cold], [fever], [duration of fever], for example, are represented as *z*_1_, *z*_2_, *z*_3_:

(4) $$\begin{array}{c} \begin{array}{c} z_{1}=\left(q,a\right)=\left(Fear\;of\;cold?,Fear\;of\;cold\right),\\ z_{2}=\left(q,a\right)=\left(Fever?,Feverish\right),\\ z_{3}=\left(q,a\right)=\left(Doesitlastlongorshort?,Short\;duration\right). \end{array} \end{array}$$

Syndrome *h* is represented as a collection of *n* symptoms: *h*={*z*_*i*_*|i*=1,2,…, *n*}, which includes both the names of the symptoms and their relationships. For example, the syndrome [syndrome of internal and external excess-cold] is represented by three symptoms: *h*={*z*_*i*_*|i*=1,2,3}, and the inquiry sequence is symptom *z*_1_ first, followed by symptom *z*_2_, and then symptom *z*_3_. In other words, the consultation's question is contextual.

#### 3.2.3. Inquiry Knowledge Base

The Ten Brief Inquiries summarizes TCM's norms and standards for the content and sequence of the inquiry [34]. The “Ten Inquiries” reads: inquire first about the cold and heat, then about the sweat; Third for the head and body, and fourth for stool and urine; Fifth for diet, and sixth for chest; Seventh for eyes and ears, and eighth for taste; Ninth for the vessel, and tenth for sniffing [35]. By classifying the contents of the inquiry according to the Ten Brief Inquiries, the order of the distinct categories is decided. The question-answer pairs are grouped into 13 categories: cold and heat, sweat, pain, taste, ears, eyes, chest, hypochondrium, stomach and abdomen, sleep, thirst, appetite, stool, and urine, and the order of the question-answer pairs for each category are determined by the corresponding content of the Ten Brief Inquiries. Question-answer pairs in the same category are logically ranked, and then all questions and answers are numbered sequentially so that each has unique, ordered IDs.

Inquiry knowledge bas*eD* = *H* ∪ *Q*, where *H* is inquiry syndrome base, *Q* is question base for inquiry. *H* = {*h*_*i*_*|i* = 1,2,…, *n*}, where *h*_*i*_ is the syndrome. *q* = {(*q*_*i*_, *s*_*i*_)*|i* = 1,2,…, *n*}, where *q*_*i*_ is question and *s*_*i*_ is the candidate answer for the user to choose from.

Table 1 depicts the question base. A sequence of question-answer pairs can be used to describe a syndrome, and their sequential order can be determined using their IDs. We connect the last question-answer pair in the sequence with the syndrome, so the set of question-answer pairs involved in each syndrome can be queried. The following question number is indicated after each question-answer pair, as shown in the last column of Table 1. If the question is the last in a series of question-answer pairs regarding a particular syndrome, it is followed by the syndrome's name.

#### 3.2.4. Inquiry Reasoning Model

Client-server architecture is used to implement the inquiry reasoning model.

- Step 1. The candidate syndromes to be identified are entered into the client, which sends the candidate syndromes to the server and requests the Q&A list, as illustrated in Figure 2. The server receives the request, searches the inquiry syndrome base for the symptoms of each candidate syndrome, retrieves the corresponding question based on the symptom, then searches the question base for candidate answers to the question, and finally organizes the questions. Their candidate answers into a list in order, removing duplicate questions to form a Q&A list, and returns it to the client.
- Step 2. After receiving the Q&A list, the client interacts with the patient. For each item on the Q&A list, the patient is given a question and the candidate answers, and he or she must pick the one that best describes his or her condition. The client then sends the patient's symptoms and candidate syndromes to the server, which differentiates the syndromes.
- Step 3. The server completes the syndrome differentiation procedure after receiving the request, as illustrated in Figure 3. The server calls the SDM interface to identify candidate syndromes, which searches the inquiry syndrome base for each candidate syndrome's symptom set and compares it to the patient's symptoms. Candidate syndromes that fit the matching criteria are confirmed and rated in order of matching degree, with the primary syndrome having the highest degree. The confirmed syndromes are returned to the client by the server.

## 4. Results and Discussion

### 4.1. Evaluation Criteria

The proposed method is evaluated in terms of the quality of the generated question-answer pairs, the accuracy of model identification, and the average number of questions. Three TCM specialists perform a manual evaluation on a scale of 1 to 5, each indicating highly unreasonable, less unreasonable, reasonable, incredibly reasonable, and perfectly consistent. Random sampling is used to imitate candidate syndromes initially identified using inspection, auscultation, and palpation. We randomly select two or three syndromes from the inquiry syndrome base as a candidate syndrome set, repeating the process ten times to obtain 20 sets. Feeding these candidate syndromes sets into our model one at a time, and the model generates a list of targeted questions and responses for interaction with the patient. We record the number of questions generated by the model for each set. One answer is chosen randomly from the candidate answers to imitate the symptoms after contact with the patient. The model returns the identification results after entering the candidate syndrome set and the patient's symptoms.

#### 4.1.1. The Quality of the Generated Question-Answer Pairs

TCM specialists separately grade each set of candidate syndromes and the Q&A list generated by the model on whether the questions generated could identify the candidate syndromes. We average the ratings of three experts to determine the quality of the generated question-answer pairs. For example, in Table 2, the model creates three questions and answers to identify the candidate syndromes” syndrome of wind and cold and dampness impediment, syndrome of cold and dampness invading the waist” with the expert scoring each question and response separately. Expert 1 considers that the first question and response can identify possible syndromes and that the question is reasonable. Thus, the first question receives a score of 3, and the same goes for the subsequent questions and responses.

#### 4.1.2. The Accuracy of Model Identification

The outcome of the syndrome differentiation is graded based on whether it is compatible with the expert's diagnosis; The closer they are, the higher the score. The model's accuracy is determined by averaging the three experts' scores.  Table 3 shows an example of the model's score for syndrome differentiation. TCM expert 1 gives the model a five because he considers the results consistent with his judgment.

#### 4.1.3. The Average Number of Questions

The model will generate a series of targeted question-answer pairs to identify candidate syndromes. We want to keep the number of pairs as small as possible while ensuring the identification results' accuracy. The fewer the pairs generated, the more consistent the questions asked by the model are with the core symptoms of the candidate syndromes. We separate validation data into two syndrome series and three syndrome series, each with ten sets of candidate syndromes. The average number of question-answer pairs generated by the model on each of the two series is determined as the average number of questions.

### 4.2. Analysis and Discussion

Figures 4 and 5 depict the three experts' grading of the model-generated questions, with the horizontal coordinates representing the ten randomly selected sets and the vertical coordinates reflecting the scores. Each set's score is the average of the questions within it. The three mean lines depict the average scores of three experts for all questions. Although the experts' assessments for the same set of questions varied, the overall scores are high, showing that the questions generated by the model are valid, accurate, relevant, and distinctive. Furthermore, expert 2 scores higher, showing that the model-generated questions are more closely aligned with his diagnostic thinking.

Figures 6 and 7 depict each expert's scoring of the model identification results. The horizontal coordinates reflect the sets, the vertical coordinates represent the scores, and the mean line represents the average scores. Sets 5, 6, and 7 have lower generated question scores and lower identification results, according to Figures 4 and 6. In contrast, the scores of generated questions and recognition results in the rest of the sets are mostly positively correlated, except in set 4, where the generated question scores are higher but the identification results are lower. Figures 5 and 7 show that the scores of generated questions in groups 4, 5, and 10 were lower than the scores of identification results. Except for group 5, where the scores of generated questions are higher, and the identification results are lower, the scores of generated questions and recognition results in the other groups are positively correlated. It demonstrates that the quality of the generated question-answer pairs affects the accuracy of the subsequent syndrome identification. Expert 2 gives the model a higher score than the other two experts, and the difference in scores between Expert 1 and Expert 3 is smaller. We guess experts specialize in different areas of TCM and have different diagnostic styles. The model's diagnostic style is more similar to Expert 2's and Expert 1's more similar to Expert 3's.

We further analyze the cases where questions' scores are high while identification results' scores are low. The symptoms that should gain through interaction with the patient are randomized after the model generates the question-answer pairs. The randomized symptoms are sometimes ineffective in identifying the candidate syndromes. Furthermore, each question in the experiment will select a response randomly as a symptom, which may not always correspond to the actual scenario. In practice, the patient may answer “none” to the issue-related symptom, and the symptom returned to the model will not include any response to the problem. Both factors lead to high scores for generated question-answer pairs and poor scores for identification results.

Using arithmetic averaging to average the scores of all experts on the model, Table 4 displays the results. After deleting one of the highest and one of the lowest scores, defining the average score as the trim mean. For the two- and three-candidate syndromes series, the scores for the produced question and the identification outcomes are above 3, showing that our approach creates high-quality questions with high identification accuracy. To identify two syndromes, the model requires an average of 4.6 questions, and for three syndromes, it takes an average of 6.4 questions. The number of questions required here is related to the model's recognition capacity. The model only requires a few questions, suggesting that the generated questions are targeted. The number of questions will be lowered further as the model's accuracy increases.

## 5. Conclusion

We develop a new TCM consultation knowledge representation method and propose a consultation-based syndrome differentiation model to address two challenges in intelligent TCM consultation research: (1) the abstract nature of TCM knowledge and (2) the scarcity of TCM consultation data. Our model identifies candidate syndromes obtained through inspection, auscultation, and olfaction by simulating inquiry. The model creates targeted question-answer pairs first, interacts with the patient next, and eventually identifies the patient's actual syndromes. We introduce manual evaluation and assess the model's effectiveness regarding the quality of the generated question-answer pairs, the accuracy of model identification, and the average number of questions. The evaluation results are also thoroughly examined and discussed. The findings suggest that our approach is capable of correctly identifying the syndromes. Furthermore, question-answer pairs generated by the model are relevant, accurate, and efficient.

The current study, while yielding some significant results, has several limitations. The SDM covers hundreds of common syndromes and works well in most cases but may be limited for less frequent syndromes and lacks generalization. In the future, we will continuously collect data from enlarging the TCM consultation datasets and combine the current method with deep learning models. In addition, we will incorporate a knowledge graph of syndromes and syndromes to improve the accuracy and reduce the number of questions.

## Figures and Tables

**Figure 1:** The correct diagnosis must be made based on deduction by the four diagnosis techniques: inspection, auscultation, interrogation, and palpation.

**Figure 2:** Based on the candidate syndrome, deduce the Q&A list.

**Figure 3:** Syndrome differentiation.

**Figure 4:** Score of generated questions for “two candidate syndromes serial”.

**Figure 5:** Score of generated questions for “three candidate syndromes serial”.

**Figure 6:** Score of identification results for “two candidate syndromes serial”.

**Figure 7:** Score of identification results for “three candidate syndromes serial.”

**Table 1:** Example of question base.

Question no.	Question	Answer no.	Answer	Next
1	Fear of cold?	A1	Fear of cold	2
		A2	No fear of cold	2

2	Fever?	A3	Fever	3
		A4	No fever	3

3	Does it last long or short?	A5	Long duration	Yang deficiency
		A6	Short duration	Pattern of internal and external excess-cold

**Table 2:** Example of rating the generated questions and answers.

Candidate syndromes	Questions	Answers	Score
Syndrome of wind and cold and dampness impediment, syndrome of cold and dampness invading the waist	Which part of the body is in pain?	Headache	3
		Chest pain	
		Flank pain	
		Stomach duct pain	
		Lumbago	
		Abdominal pain	
		Back pain	
		Pain in limbs	
		Body pain	
	What is the pain in the waist?	Frequent soreness	3
		Cold pain and feeling heavy worsens on rainy days	
		Stabbing pain	
		Pain extending to lower limbs	
		Sudden sharp pain	
		Pain that cannot be tilted	
	What kind of back pain is it?	Pain that cannot be tilted	3
		Nape back pain	
		Fixed or scurrying pain rises when exposed to wind-cold	

**Table 3:** Example of the model's score for syndrome differentiation.

Candidate syndromes	Questions	Answers	Symptoms of the patient	Differentiation result	Score
Syndrome of wind and cold and dampness impediment, syndrome of cold and dampness invading the waist	Which part of the body is in pain?	Headache	Lumbago	Syndrome of cold and dampness invading the waist	5
		Chest pain			
		Flank pain			
		Stomach duct pain			
		Lumbago			
		Abdominal pain			
		Back pain			
		Pain in limbs			
		Body pain			
	What is the pain in the waist?	Frequent soreness	Cold pain and feeling heavy worsens on rainy days		
		Cold pain and feeling heavy worsens on rainy days			
		Stabbing pain			
		Pain extending to lower limbs			
		Sudden sharp pain			
		Pain that cannot be tilted			
	What kind of back pain is it?	Pain that cannot be tilted	Fixed or scurrying pain rises when exposed to wind-cold		
		Nape back pain			
		Fixed or scurrying pain rises when exposed to wind-cold			

**Table 4:** Expert evaluation results in summary.

Serial	2 candidate syndromes	3 candidate syndromes
Average score of the generated questions	3.82	3.90
Average score of the identification results	3.30	3.43
Trim mean of the generated questions	3.79	3.95
Trim mean of the identification results	3.42	3.46
The average number of questions	4.60	6.40

## Data Availability

The data used to support the findings of this study are available from the corresponding author upon request.
